The article "Comparison between an Acrylic Splint Herbst and an Acrylic Splint Miniscrew-Herbst for Mandibular Incisors Proclination Control" was published in 2014. Journal: Int J Dent.

# Comparison between an Acrylic Splint Herbst and an Acrylic Splint Miniscrew-Herbst for Mandibular Incisors Proclination Control

**DOI:** 10.1155/2014/173187

**Published:** 2014-05-19

**Authors:** Antonio Manni, Marco Pasini, Laura Mazzotta, Sabrina Mutinelli, Claudio Nuzzo, Felice Roberto Grassi, Mauro Cozzani

**Affiliations:** ^1^Private Practice Lecce, Via Giacobina, 6 Racale, 73055 Lecce, Italy; ^2^Private Practice Massa, Viale Roma 213, 54100 Massa, Italy; ^3^Orthodontic Department, Cagliari University, via Binaghi 4, 09121 Cagliari, Italy; ^4^Private Practice Trento, Viale Roma 20, 38066 Riva del Garda, Italy; ^5^Hospital Vito Fazzi, Piazza F. Muratore Snc, 73100 Lecce, Italy; ^6^Interdisciplinary Department of Medicine, Università Aldo Moro, Piazza Umberto I, 70121 Bari, Italy; ^7^UO Odontoiatria (Istituto Giannina Gaslini), Private Practice, Via Fontevivo 21N, 19125 La Spezia, Italy

## Abstract

*Aim*. The aim of this study is to compare dental and skeletal effects produced by an acrylic splint Herbst with and without skeletal anchorage for correction of dental class II malocclusion. *Methods*. The test group was formed by 14 patients that were treated with an acrylic splint miniscrew-Herbst; miniscrews were placed between mandibular second premolars and first molars; controls also consisted of 14 subjects that were treated with an acrylic splint Herbst and no miniscrews. Cephalometric measurements before and after Herbst treatment were compared. The value of *α* for significance was set at 0.05. *Results*. All subjects from both groups were successfully treated to a bilateral Class I relationship; mean treatment time was 8,1 months in the test group and 7.8 in the controls. Several variables did not have a statistical significant difference between the two groups. Some of the variables, instead, presented a significant difference such as incisor flaring, mandibular bone base position, and skeletal discrepancy. *Conclusions*. This study showed that the Herbst appliance associated to miniscrews allowed a better control of the incisor flaring with a greater mandibular skeletal effect.

## 1. Background

The Herbst appliance is largely used in orthodontics for correction of class II malocclusions and among the different types of functional appliances it has been reported to be one of the most efficient [1, 2]; it has become increasingly popular because it does not need patient compliance and because the treatment time required is short, therefore willingly accepted by patients [3, 4]. Its effects are both dental and skeletal and include a posterior displacement of the upper dental arch, an anterior displacement of the lower dental arch, a reduced sagittal growth of the maxilla, and an enhanced sagittal growth of the mandible. It should be kept in mind that these skeletal effects vary among subjects, between sexes, and within treatment times [4]. Also it is well known that Herbst treatments cause a proclination of lower incisors due to anchorage loss [5, 6] in different amounts relative to the type of Herbst used; various modifications of the original Herbst, such as the use of class III elastics, reduced cast splints, and total cast splints, have been proposed, but none has been able to completely stop the proclination of mandibular incisors [7, 8]. Today there is in literature only one study that showed a reduction of lower incisor flaring by using acrylic splint Herbst appliances [9] to 2,5 degrees in a 10-month treatment period.

The introduction of skeletal anchorage in orthodontics not only has allowed the simplification of many procedures conventionally employed for the control of anchorage, but also has reduced the undesirable effects of many appliances [10]. Moreover, miniscrews present many advantages, including low cost, low invasive insertion procedures and great versatility. Many authors have demonstrated that they can be used as a successful source of anchorage during orthodontic therapy [11, 12]. The possibility of combining Herbst appliance with skeletal anchorage has been previously described in literature in two studies [13, 14] and both showed a reduction of mandibular incisors flaring. However, there is no case-control study in literature that thoroughly analyses the effects of a miniscrew combined Herbst. Therefore, the aim of this study is to compare dental and skeletal effects produced by an acrylic splint Herbst with and without skeletal anchorage for correction of dental class II malocclusion.

## 2. Methods

Inclusion criteria for this retrospective study were: patients who could benefit from a Herbst treatment, that had a bilateral Angle Class II division 1 malocclusion (≥1/2 cusp width), who were in permanent or late mixed dentition, and whose parents had signed an informed consent form. Exclusion criteria were: poor oral hygiene and motivation, tooth agenesis or premature loss of permanent teeth, presence of second molars, transverse or vertical discrepancies, and incomplete available records. All the patients were evaluated and treated by a single operator (A.M.) and divided into two groups.

- Group 1 (tests) consisted of 14 subjects that were consecutively treated with an acrylic splint miniscrew-Herbst; it included 6 males and 8 females with a mean age of 12,36 ± 1,5 years. Miniscrews were placed between mandibular second premolars and first molars in the attached gingiva [15] and were ligated with elastic chains (Memory Chain—American Orthodontics ©, Sheboygan, WI). During treatment, elastic chains have been replaced every 30 to 60 days.
- Group 2 (controls) consisted of 14 subjects that were treated with an acrylic splint Herbst and no miniscrews; the group included 6 males and 8 females with a mean age of 12,28 ± 1,07 years; subjects were chosen by pairing the data to create a group that was homogeneous with the cases for what concerned the age and sex variables.

The miniscrews employed (M.A.S., Micerium, Avegno, Italy) were in titanium, 11 mm long, and shaped like a truncated cone with a diameter of 1.5 mm or 1.3 mm (according to the bone level) at the point and 2.2 mm at the neck. The shank of the screws measured 1 mm in diameter; the threaded part had a length of 9–11 mm and the heads featured a hexagonal slot that could house the head of the screwdriver or a contra-angle handpiece.

Before the insertion of the miniscrew, each patient rinsed his mouth with 0.1% chlorhexidine gluconate solution; predrilling was carried out and the miniscrews were inserted by means of a manual screwdriver.

Elastic ligatures (100 g) linked the miniscrews to metallic buttons bonded to the lower canines of each side (Figure 1). Lateral cephalometrics were obtained from all patients before (T1) and at the end (T2) of the Herbst treatment to evaluate the outcome of the orthodontic therapy. The SO-analysis of Pancherz (analysis of changes in sagittal occlusion) [16] was carried out for each patient at T0 and at T1 to analyze skeletal and dental changes (Figure 2).

The OL (Occlusal Line) and the OLp (Occlusal Line Perpendicular) were transferred from T1 to T2 cephalometrics by superimposition of the radiographs on the stable bone structures of the anterior cranial base. Furthermore, other parameters that are not considered in Pancherz SO-analysis were included, such as mandibular incisor proclination (Ii/GoMe) and skeletal divergence (SN/GoMe); variables considered are shown in Table 1.

All linear and angular measurements were taken to the nearest 0.5 mm and 0.5 degrees, respectively. All these measurements were performed twice, with a seven day interval between the two recordings, in order to calculate Dahlberg's formula [17]: the method error resulted to be less than 1 mm, for linear measurements, and less than 1° for angular measurements.

## 3. Statistical Analysis

Measurements of the two groups were compared using the unpaired *t* test for normally distributed variables and the Wilcoxson test when the assumption of normality was not complied with. The variation between T1 and T2 for each group was evaluated with the *t*-test for paired data; the value of *α* for significance was set at 0.05.

## 4. Results

All subjects from both groups have been successfully treated to a bilateral Class I relationship. The mean treatment time (from T1 to T2) in the miniscrew group was 8.1 ± 1.7 months, while in the control group it was 7,8 ± 1.1; four miniscrews had to be replaced because of their mobility during treatment.

At baseline, groups presented statistical significant differences: patients treated with the miniscrew Herbst had a greater mandibular incisor proclinationat pretreatment being the mean value in the control group 95.4 ± 4.1° and in the test group 100.5 ± 6.0° (*P* = 0.0149). Also, the control group was composed by both more maxillary and mandibular retruded patients and by subjects with a shorter mandible than the skeletal anchored group patients. As a matter of fact, mean A/OLp (maxillary bone base) values at T1 in the control group was 76.5 ± 1.0 mm while in the test group was 79.5 ± 1.0 mm (*P* = 0.0401). Also at T1 the mean value of Pg/OLp (mandibular bone base) in the control group was 78.6 ± 3.9 mm while in the miniscrew group was 82.4 ± 5.1 mm (*P* = 0.0406) and the mean value of Ar/OLp + Pg/OLp at T1 (mandibular length) in the control group was 86.9 ± 4.5 mm while in the miniscrew group was 90.8 ± 4.8 mm (*P* = 0.0372). In addition, patients in the control group presented mandibular incisors (Ii) in a more lingualized position (T1 mean value in the control group: 77.0 ± 1.0 mm; test group: 80.3 ± 1.1 mm; *P* = 0,037).

A few variables did not undergo any variation in both groups: changes in maxillary bone base were nonsignificant (*P* = 0.266 for the control group and 0.728 for the test group) together with condyle position (*P* = 0.385 for the control group and *P* = 0.076 for the test group) and skeletal divergence (*P* = 0.788 for the control group and *P* = 0.189 for the test group).

Also, maxillary incisors had a slight variation: statistical analysis showed a difference between the groups at T2 (*P* = 0.0146) but not at baseline (*P* = 0.1004). However this difference is clinically not relevant and statistically negligible.

Some of the variables on the contrary changed in both groups; skeletal class, for example, improved significantly in tests (T2-T1: 2.6°) and in controls (T2-T1: 1.6°). Mandibular incisors also reached a more buccal position both in the control (T2-T1: −2.4 mm) and in the test groups (T2-T1: −3.4 mm). Overjet also decreased in a similar way both in controls (T2-T1: 3.1 mm) and in tests (T2-T1: 2.5 mm). In addition mandibular molars mesialized in a statistically significant way in the control group (T2-T1: −2.1 mm) and in the test group (T2-T1: −4.1 mm). Molar relationship (which is the difference between the linear measurement of the maxillary molar and the mandibular molar; Ms/Olp − Mi/Olp;) improved since mean difference T2-T1 resulted to be 5.4 mm in controls and 5 mm in tests.

Several values underwent changes only in one group: statistical analysis showed, for example, that variations of the mandibular bone base were significant only in the group with skeletal anchorage (T2-T1: −3.4 mm; *P* = 0.002). The control group had a mean change of −1.6 mm that resulted to be nonsignificant (*P* = 0.257).

Also, the group treated with skeletal anchorage underwent a significant increase in mandibular length (T2-T1: −4.6 mm), while the control group did not significantly change (T2-T1: −0.9; *P* = 0.263). Skeletal discrepancy was reduced more in the group with skeletal anchorage because of pogonion advancement: A/Olp − Pg/Olp had a mean change of 3.6 mm in the test group (*P* = 0.0001) and of 0.3 mm in the control group (*P* = 0.612). Maxillary molars underwent a statistically significant distalization (T2-T1: 3.2 mm; *P* = 0.002) only in the control group. Molar distalization in the test group resulted to be nonsignificant (*P* = 0.111). Statistical analysis also clearly showed that mandibular incisor proclination increased in a clinically relevant way in the control group patients, while in the skeletal anchorage group no proclination was observed. As a matter of fact, the mean difference in the control group was 7.5 degrees (*P* = 0.0001) whereas in the tests it resulted to be 0.6 degrees (*P* = 0.713).

All results are shown in Tables 2 and 3.

## 5. Discussion

Our results show that both treatments are effective in correcting class II malocclusion; in fact a bilateral molar class I was achieved in all patients. In both groups it was noticed a significant decrease of the overjet with a mesial movement of mandibular molars and no variation of the maxillary bone base position. Also, in agreement with other studies found in literature [18, 19], skeletal divergence was not affected by the treatment.

Some of the cephalometric variables, however, underwent a statistical change only in the test group: miniscrew Herbst treatment seems to have a greater skeletal effect on the mandible since only in this group mandibular bone base (Pg/OLp) advanced significantly and mandibular length (Ar/OLp + Pg/OLP) increased consistently; as a matter of fact, a reduction of the skeletal discrepancy could be observed only in this group.

Molar relationship (MS/OLp − Mi/OLp) changed similarly in both groups; yet, in the control group the reduction is due to a combination between the distalization of the upper molar and a mesial movement of the mandibular molar, while in the test group it is due just to mandibular molar advancement.

Above all, what is showed in this study is that the combination of Herbst and miniscrews allowed a significantly better control of mandibular incisor proclination, in comparison with the control patients: incisor flaring after treatment in the test group resulted to be 0.6°. This is in agreement with what is showed by Luzi et al. in their case report [13] since they showed a proclination of 1°; however, they used a cast splint Herbst and 012” stainless steel ligatures to ligate miniscrews. On the contrary, incisor proclination after treatment in the control group had an increase of 7.5°; this value is slightly lower if compared to values found in literature: studies report mean values of lower incisor proclination of 8.9° [20] and of 10.8° [21] after the use of the total mandibular cast splint Herbst. von Bremen et al. [22] showed a mean proclination of 11.8° and 9.3°, with reduced and total mandibular cast splints Herbst, respectively. Other studies also have shown similar values of incisor proclination, even when combining the Herbst appliance with a lingual fixed appliance [23–25]. In this study an acrylic splint Herbst was used because in literature it has been reported to have a better mandibular incisor proclination control [9]; as a matter of fact, mean values of incisor flaring are slightly lower than values founded in literature; yet, they are higher than the ones reported by Valant and Sinclair [9]. In any case, it seems that the only way to fully control the anchorage loss that occurs when using a Herbst appliance may be the use of miniscrews.

According to our results, it may seem that a better mandibular incisor proclination control would allow a slightly mesial displacement of the mandible and a greater skeletal effect. This found a confirmation in literature only in one animal study [26]: an evaluation of the effects of mandibular advancement plus the inhibition of lower incisor movement on mandibular growth in rats showed that mandibular growth was accelerated before and during the pubertal period. Moreover, Valant and Sinclair's study [9] showed a greater control of incisor flaring combined to a greater mandible growth and a minimal headgear effect.

Also, concerning mandibular incisors, it may seem contradictory to find out that treatment result revealed a larger (however, not significant) labial displacement of the teeth (Ii/OLp) in the test group (3.4 mm) than in the control group (2.4 mm). The opposite was true when measuring the inclination changes of the teeth as in the test group the incisors were significantly less proclined than in the control group. However, in the test group an advancement of the pogonion was observed, which implies a labial displacement of mandibular incisors.

The two groups showed differences also for what concerns forces on maxillary molars: the group treated with miniscrews showed no distalizing effect, which instead was present in the control group; we are conducting a new research to investigate this effect.

In this study, the two groups were paired to be similar for age and sex; at baseline, however, groups presented statistical significant differences: patients treated with the miniscrew Herbst at pretreatment had a greater mandibular incisor proclination; however, with miniscrews no anchorage loss was found. Also, the control group was composed by both more maxillary and mandibular retruded patients and had a shorter mandible and at the end of treatment maxillary bone base had remained stable in both groups while mandibular bone base and mandibular length had increased only in the test group.

In addition, at T1 patients in the control group presented mandibular incisors in a more lingualized position; mandibular incisors reached at the end of treatment a more buccal position in both groups; however, statistic data have shown that in the control group it was due to incisor flaring while in the test group it was due to mandibular advancement.

## 6. Conclusion

This preliminary study showed that an acrylic splint Herbst appliance associated to miniscrews could allow a better control of the incisor flaring with a greater mandibular skeletal effect. More studies are needed to increase the sample size and to have more homogeneous groups.

## Figures and Tables

**Figure 1:** Acrylic splint miniscrew Herbst; elastic ligatures (100 g) linked the miniscrews to metallic buttons bonded to the lower canines of each side.

**Figure 2:** Modified SO-Pancherz analysis: measuring landmarks and distances.

**Table 1:** Cephalometric variables analysed and their description.

(1) Maxillary bone base	A/Olp: distance from point A to the Olp line (mm)
(2) Mandibular bone base	Pg/Olp: distance from point Pg to the Olp line (mm)
(3) Mandibular length	Ar/Olp + Pg/Olp: condile plus mandibular base (mm)
(4) Skeletal discrepancy	A/Olp − Pg/Olp: maxillary bone base minus mandibular bone base (mm)
(5) Skeletal class	AN/NPg: angle formed by the lines AN and NPg (degrees)
(6) Skeletal divergence	SN/GoMe: angle formed by the lines SN and GoMe (degrees)
(7) Maxillary incisor	Is/Olp: distance from point Is to the Olp line (mm)
(8) Mandibular incisor	Ii: distance from point Ii to the Olp line (mm)
(9) Mandibular incisor proclination	Ii/GoMe: angle formed by the mandibular incisor axis and the mandibular plane (GoMe); (degrees)
(10) Overjet	Is/Olp − Ii/Olp: maxillary incisor minus mandibular incisor (mm)
(11) Maxillary molar	Ms/Olp; Ms: distance from point Ms to the Olp line (mm)
(12) Mandibular molar	Mi/Olp: distance from point Mi to the Olp line (mm)
(13) Molar relationship	Ms/Olp − Mi/Olp: maxillary molar minus mandibular molar (mm)
(14) Condyle position	Ar/Olp: distance from point Ar to the Olp line (mm)

**Table 2:** *t*-test for unpaired data and Wicoxson rank sum test. Values at T1 and T2 and differences between groups.

Variable	Standard group (*n* = 14)		Miniscrew group (*n* = 14)		Difference between groups			
	T1 [mean (SD)]	T2 [mean (SD)]	T1 [mean (SD)]	T2 [mean (SD)]	T1 [mean (95% CI)]	*P*	T2 [mean (95% CI)]	*P*
A/Olp, mm	76.5 (1.0)	75.8 (1.0)	79.5 (1.0)	79.3 (1.1)	0.96 (0.93 to 1.0)	0.0401	0.96 (0.92 to 1.0)	0.0335
Pg/Olp, mm	76.6 (3.3)	78.1 (1.5)	82.4 (5.1)	85.8 (5.7)	−5.8 (−9.2 to −2.4)	0.002	−7.6 (−12.0 to −3.2)	0.0014
Is/Olp, mm	83.2 (1.0)	82.4 (1.1)	85.9 (1.1)	86.9 (1.1)	0.97 (0.9 to 1.0)	0.1004	0.95 (0.91 to 0.99)	0.0146
Ii/Olp, mm	77.0 (1.0)	79.3 (1.1)	80.3 (1.1)	83.7 (1.1)	0.96 (0.92 to 1.00)	0.037	0.95 (0.91 to 0.99)	0.0164
Ms/Olp, mm	51.1 (2.6)	49.9 (4.0)	54.6 (4.6)	53.8 (4.8)	−3.5 (−6.4 to −0.6)	0.021	−3.85 (−7.3 to 0.4)	0.0299
Mi/Olp, mm	51.1 (2.6)	53.3 (3.7)	53.6 (5.3)	57.7 (6.4)	−2.4 (−5.7 to 0.9)	0.1378	−4.4 (−8.5 to −0.3)	0.0361
A/Olp − Pg/Olp, mm	−0.1 (3.7)	−2.3 (3.8)	−2.7 (3.0)	−6.4 (3.2)	0.7 (−1.9 to 3.3)	0.5808	4.1 (1.3 to 6.8)	0.005
Is/Olp − Ii/Olp, mm	6.2 (2.2)	3.1 (1.5)	5.6 (1.9)	3.1 (0.9)	0.6 (−1.1 to 2.2)	0.4759	−0.1 (−1.0 to 0.9)	0.881
Ms/Olp − Mi/Olp, mm	2 (2)	−3.4 (1.7)	1.1 (1.7)	−3.9 (3.4)	0.9 (−0.5 to 2.4)	0.2004	0.6 (−1.5 to +2.7)	0.5789
Ar/Olp, mm	8.3 (4.2)	8.9 (3.3)	8.4 (3.2)	9.6 (4.2)	−0.1 (−3.0 to 2.8)	0.92	−0.6 (−3.6 to 2.3)	0.6579
Ar/Olp + Pg/Olp, mm	86.9 (4.5)	87.8 (5.5)	90.8 (4.8)	95.4 (5.9)	−3.9 (−7.5 to −0.25)	0.0372	−7.6 (−12.0 to −3.2)	0.0015
Ii/GoMe, degrees	95.4 (4.1)	102.9 (8.0)	100.5 (6.0)	101.1 (7.1)	−5.1 (−9.1 to −1.1)	0.0149	1.9 (−4.0 to 7.6)	0.5228
AN/NPg, degrees	5 (2)^*∗*^	3 (1)^*∗*^	4 (3)^*∗*^	2.5 (3)	1 (6)^*∗*^	0.8162^*∗∗*^	0.5 (4)^*∗*^	0.3979^*∗∗*^
SN/GoMe, degrees	31.6 (6.0)	31.9 (7.2)	33.5 (5.1)	32.6 (5.2)	−1.9 (−6.2 to 2.5)	0.3864	−0.8 (−5.7 to 4.1)	0.7435

*Median and interquatile range for not normally distributed data.

**Wilcoxon rank sum test.

**Table 3:** *t*-test for paired and unpaired data: difference from T1 to T2.

Variable	Standard group (*n* = 14)		Miniscrew group (*n* = 14)		Difference between groups	
	T2-T1 [mean (95% CI)]	*P*	T2-T1 [mean (95% CI)]	*P*	Mean (95% CI)	*P*
A/Olp, mm	2.8 (1.3 to 4.4)	0.003	0.2 (−1.1 to 1.5)	0.728	2.6 (0.6 to 4.6)	0.015
Pg/Olp, mm	−1.6 (−4.4 to 1.3)	0.257	−3.4 (−5.3 to −1.6)	0.002	1.9 (1.8 to 6.1)	0.253
Is/Olp, mm	0.8 (−1.2 to 2.8)	0.42	−0.9 (−2.6 to 0.8)	0.26	1.7 (−0.8 to 4.2)	0.1752
Ii/Olp, mm	−2.4 (−3.9 to −0.8)	0.007	−3.4 (−4.9 to −1.9)	0.0001	1.1 (−1.0 to 3.2)	0.2998
Ms/Olp, mm	3.2 (1.8 to 4.6)	0.002	0.9 (−0.2 to 1.9)	0.111	2.4 (0.7 to 4.0)	0.0075
Mi/Olp, mm	−2.1 (−3.8 to −0.5)	0.016	−4.1 (−6.1 to −2.2)	0.001	2.0 (−0.5 to 4.5)	0.1072
A/Olp − Pg/Olp, mm	0.3 (−0.9 to 1.5)	0.612	3.6 (2.2 to 5.1)	0.0001	−3.4 (−5.0 to −1.6)	0.0007
Ar/Olp, mm	−0.6 (−2.2 to 0.9)	0.385	−1.1 (−2.4 to 0.1)	0.076	0.5 (−1.4 to 2.4)	0.5948
Ar/Olp + Pg/Olp, mm	−0.9 (−2.4 to 0.7)	0.263	−4.6 (−6.4 to −2.8)	0.0001	3.7 (1.5 to 6.0)	0.0024
Ii/GoMe, degrees	−7.5 (−10.7 to −4.3)	0.0001	−0.6 (−3.9 to 2.7)	0.713	−6.9 (−11.3 to −2.6)	0.0031
Ms/Olp − Mi/Olp, mm	5.4 (3.6 to 7.1)	0.0001	5 (2.9 to 7.1)	0.0001	0.4 (−2.2 to 2.9)	0.7784
SN/GoMe, degrees	−0.2 (−1.9 to 1.5)	0.788	0.9 (−0.5 to 2.2)	0.189	−1.1 (−3.1 to 1.0)	0.2913
Is/Olp − Ii/Olp, mm	3.1 (2.0 to 4.3)	0.0001	2.5 (1.4 to 3.6)	0.0001	0.6 (−0.9 to 2.2)	0.3919
AN/NPg, degrees	1.6 (0.5 to 2.7)	0.007	2.6 (1.9 to 3.3)	0.0001	−0.9 (−2.2 to 0.3)	0.137
